The article "Effective Image Processing and Segmentation-Based Machine Learning Techniques for Diagnosis of Breast Cancer" was retracted in 2023. Reasons: signs of a paper mill; suspected computer-generated content; unreliable results or conclusions; concerns about the data.

# Effective Image Processing and Segmentation-Based Machine Learning Techniques for Diagnosis of Breast Cancer

**DOI:** 10.1155/2022/6841334

**Published:** 2022-04-08

**Authors:** Sushovan Chaudhury, Alla Naveen Krishna, Suneet Gupta, K. Sakthidasan Sankaran, Samiullah Khan, Kartik Sau, Abhishek Raghuvanshi, F. Sammy

**Affiliations:** ^1^University of Engineering and Management, Kolkata, India; ^2^Mechanical Engineering Department, Institute of Aeronautical Engineering, Hyderabad, India; ^3^Department of CSE, School of Engineering and Technology, Mody University, Lakshmangarh, Rajasthan, India; ^4^Department of ECE, Hindustan Institute of Technology and Science, Chennai, India; ^5^Department of Maths, Stat & Computer Science, The University of Agriculture, Pakistan; ^6^University of Engineering and Management, Kolkata, West Bengal, India; ^7^Mahakal Institute of Technology, Ujjain, India; ^8^Department of Information Technology, Dambi Dollo University, Dembi Dolo, Welega, Ethiopia

## Abstract

Breast cancer is the second leading cause of death among women, behind only heart disease. However, despite the high incidence and mortality rates associated with breast cancer, it is still unclear as to what is responsible for its development in the first place. The prevention of breast cancer is not possible with any of the current available methods. Patients who are diagnosed and treated for breast cancer at an early stage have a better chance of having a successful treatment and recovery. In the field of breast cancer detection, digital mammography is widely acknowledged to be a highly effective method of detecting the disease early on. We may be able to improve early detection of breast cancer with the use of image processing techniques, thereby boosting our chances of survival and treatment success. This article discusses a breast cancer image processing and machine learning framework that was developed. The input data set for this framework is a sequence of mammography images, which are used as input data. The CLAHE approach is then utilized to improve the overall quality of the photographs by means of image processing. It is called contrast restricted adaptive histogram equalization (CLAHE), and it is an improvement on the original histogram equalization technique. This aids in the removal of noise from photographs while simultaneously improving picture quality. The segmentation of images is the next step in the framework's development. An image is divided into distinct portions at this point because the pixels are labeled at this step. This assists in the identification of objects and the delineation of boundaries. To categorize these preprocessed images, techniques such as fuzzy SVM, Bayesian classifier, and random forest are employed, among others.

The article "Effective Image Processing and Segmentation-Based Machine Learning Techniques for Diagnosis of Breast Cancer" was retracted in 2023. Reasons: signs of a paper mill; suspected computer-generated content; unreliable results or conclusions; concerns about the data.

## 1. Introduction

Women are more likely than men to develop breast cancer [1, 2], but men can also develop the disease. Aside from a few minor differences, the breasts of both men and women are structurally identical to one another. There are glandular structures in the breast known as lobules that produce milk and ducts that transport the milk to the nipple, both of which are located in the chest cavity. The glandular tissue and ducts are surrounded by a ring of fat and fibrous connective tissues. There are no muscles in the breasts themselves. Lymphatic nodes are located throughout the breast and are responsible for removing excess fluid and white blood cells. Breast cancer usually begins in the lobules or ducts of the breast, but it can also begin anywhere in the breast. Fat or connective tissue can serve as a potential starting point for the procedure. Breast cancer is characterized by uncontrolled cell division, expansion, and death in the breast tissue. As a result of the uneven cell development, a lump or bulk is formed. The lumps continue to grow in size over time, until they are large enough to be felt. It is possible that the abnormal lumps are not cancerous and are instead either a benign mass or a tumor. As cancer cells continue to proliferate and disseminate, they have the potential to invade normal tissues and the lymphatic node system. Cancer can spread to other parts of the body through the lymph nodes [3].

In the last few decades, breast cancer has risen to the top of the list of the most common diseases afflicting women around the world. It is the most frequent cancer among women worldwide and the primary cause of death.

The disparity between the number of cancer cases and the number of those who survive is expanding on a regular basis, according to cancer data. As a result, early identification of breast cancer has become a top concern. Different imaging modalities such as MRI, ultrasound, and thermal imaging have become essential in the management of cancer patients for the detection and diagnosis of cancer tumors [4].

In terms of cost and reliability, mammography is the best imaging technique for detecting early signs of breast cancer. Mammographic scans can reveal masses, microcalcifications, architectural defects, and bilateral asymmetry [5].

False positives are abnormalities that appear to be cancerous but are actually harmless. In the event of a misdiagnosis, patients would have to undergo more testing and diagnostic procedures, which would add to their anxiety. Breast cancer patients can choose from a variety of treatment options, depending on the severity of their disease. Breast cancer treatment decisions are often based on a variety of factors. Patients' age, tumor size, and kind of cancer are just a few of these variables [6, 7].

The article "Effective Image Processing and Segmentation-Based Machine Learning Techniques for Diagnosis of Breast Cancer" was retracted in 2023. Reasons: signs of a paper mill; suspected computer-generated content; unreliable results or conclusions; concerns about the data.

The second biggest cause of death in women is breast cancer [8]. Despite the high incidence and mortality rates associated with breast cancer, the specific origin of the disease remains a mystery. Breast cancer cannot be prevented in any way that is currently effective. By detecting and diagnosing breast cancer at an early stage, patients have a better opportunity for successful treatment and recovery. It is well accepted that digital mammography is an effective method for detecting breast cancer. Using image processing and machine learning techniques [9, 10], we may be able to enhance early identification of breast cancer, therefore increasing our chances of survival and treatment success.

This article describes a breast cancer image processing and machine learning framework. A series of mammography pictures is employed as the input data set in this framework. Image processing is then used to increase the quality of these photos using the CLAHE method. CLAHE, or contrast limited adaptive histogram equalization, is an improvement on the original histogram equalization approach. This helps to remove noise from photos while also increasing image quality. The framework's next stage is picture segmentation. Pixels are labeled in this stage, which separates a picture into various pieces. This aids in the location of objects and boundaries. Fuzzy SVM, Bayesian classifier, and random forest approaches are used to classify these preprocessed pictures.

## 2. Literature Survey

This section contains a literature survey of various techniques used for the mammogram image preprocessing, image segmentation, and image classification in context of the breast cancer detection.

### 2.1. Survey of Image Enhancement Techniques

The probability distribution of the histogram of the mammographic image is viewed. The most information is included in the histogram's uniform distribution, according to the information theory. Therefore, the mammography data must be maximized in order to disperse the gray levels in order to create the most uniform histogram possible. While the overall dynamic range provided by adaptive histogram equalization boosts contrast in radiological pictures, small local feature gray levels vary [11].

The difference picture, which contains the image's details, is created by subtracting the original image from a blurred negative. The initial blurred image just enhances and adds to the details. Image quality improves because only the highest-frequency features are boosted, resulting in a crisper image [12].

The article "Effective Image Processing and Segmentation-Based Machine Learning Techniques for Diagnosis of Breast Cancer" was retracted in 2023. Reasons: signs of a paper mill; suspected computer-generated content; unreliable results or conclusions; concerns about the data.

In many photographs, the dominant item of interest is a small, isolated location, and the image's background does not add much to the overall interpretation. A picture's background can be reduced by subtracting a low-pass filtering version of the original image from itself in order to improve the gray level variation in the image's details. Both spine filtering and gray scale morphological processing have been used to estimate the image backdrop succeeded in accomplishing this goal [12].

An image's background can only be accurately identified if the background extraction method can adapt to the specific properties of a given image. In CLAHE, the histogram is computed only for the pixel's surrounding context. By imposing a user-specified maximum, or clip level, to the height of the local histogram and hence the maximum contrast enhancement factor, CLAHE limits the maximum contrast adjustment. This reduces the amount of noise in the final image. CLAHE is superior at enhancing tiny areas in mammography [11]. When viewed in comparison to a white background, the lesions are clearly visible. In spite of the increased visibility of both signal and noise with this approach, graininess is still evident in the photos.

In their study, authors [13] proposed ANCE using a technique known as region growth; the method creates a homogeneous area around the pixel that is being worked on. The region's contrast to its surroundings is calculated. For low-contrast regions with background pixels that have a standard deviation normalized to their mean of less than 0.1, it is possible to increase the contrast of that region by varying its intensity; however, for high-contrast regions with a variable background, this procedure of varying intensity is not possible. To calculate the contrast, ANCE uses the optical contrast definition, where the grouping of pixels is referred to as “neighborhoods,” and each pixel is assigned one. This technique improves the visibility of objects with a wide range of dimensions.

The first step in direct image enhancement is to choose an appropriate contrast measure for the image being worked on. In the past, a variety of contrast metrics have been proposed. For example, the Michelson contrast measure and the Weber contrast measure are only adequate for basic patterns and are not suitable for assessing contrast in more complicated images. Contrast measures derived in the wavelet domain were employed. A multiscale structure underpins the contrast measurement. The enhanced photos have a superior visual quality because of this method's modification of a multiscale measure that suits the human vision system. There may be instances where this contrast augmentation does not meet the standards set by multiple scales, resulting in a subpar final result. Some scales require more attention to detail than others.

The article "Effective Image Processing and Segmentation-Based Machine Learning Techniques for Diagnosis of Breast Cancer" was retracted in 2023. Reasons: signs of a paper mill; suspected computer-generated content; unreliable results or conclusions; concerns about the data.

### 2.2. Survey of Image Segmentation Techniques

The gray-level values are the basis for the adaptive histogram thresholding method. The PDF curve selects a global threshold for the entire image based on its selection. Segmenting tumors in mammograms with this procedure is rapid, easy, and effective. As a result, suspicious mass segmentation might be challenging because thick breast tissues, which may have a higher density than the suspicious masses, often overlap with the suspicious masses. By using global gray-level thresholding, it is difficult to accurately identify lesions in the mammograms. For each pixel in a specific set of nearby windows, the window-based adaptive thresholding algorithm adaptively picks the appropriate threshold. When a lesion is clearly visible, the pixels can be easily segregated since their nearby windows have a higher gray-level value. Adaptive thresholding based on multi resolution in mammograms was proposed by [14].

It was found that [14] could detect suspicious lesions in multiscale images by using a combination of two thresholding segmentations, i.e., a coarse segmentation and a fine segmentation. In order to obtain more exact segmentation findings, coarse segmentation is utilized to generate a rough representation of suspicious lesions' location. Fine segmentation is then used to refine the rough representation. The coarse segmentation is implemented using a histogram-based adaptive thresholding technique.

The *K*-means clustering technique divides the data into a predetermined number of groups. Cluster centers should be chosen at random for each cluster. The further apart these facilities are the better. In this approach, the Euclidean distance between data points and centroids is mostly utilized.

Adaptive *K*-means clustering for breast image segmentation was proposed by [15] for the detection of micro calcifications. By using this algorithm, radiologists may make a more accurate diagnosis of microcalcifications in digital mammography images by simply looking at them, and the method's detection accuracy has also improved.

*K*-means is a well-known method that can be extended to include fuzzy *C*-means [16]. Because each image pattern can be connected with every cluster using a fuzzier membership function in fuzzy *C*-means, rather than a single cluster in *K*-means, this is the main distinction.

Rough *K*-means (RKM) is a *K*-means method that utilizes rough sets [17]. The higher approximation can be considered a subset of the lower approximation, at least in theory. Boundary region refers to the area between the upper and lower approximations that contains objects from different clusters.

The article "Effective Image Processing and Segmentation-Based Machine Learning Techniques for Diagnosis of Breast Cancer" was retracted in 2023. Reasons: signs of a paper mill; suspected computer-generated content; unreliable results or conclusions; concerns about the data.

### 2.3. Survey of Image Classification Techniques

The process of picture categorization is based on the analysis of a variety of visual characteristics. Several data instances are used in the training and testing of this classification method. There will be a target value and numerous attributes for each instance in the training set.

Statistical learning theory uses the SVM as a method for teaching and learning [18]. It is based on the notion of minimizing structural risk. As a result, it reduces the bound on generalization error, which happens due to data that the learning machine does not observe during training, rather than mean square error over the data set like other machine learning algorithms. SVM performs effectively when applied to test data for this reason.

A linear classifier, a single-layer perceptron is the most basic feed forward artificial neural network. Only linearly separable sets can be used with this algorithm, which only has one neuron. In a feed-forward artificial neural network, a multilayer perceptron (MLP) has numerous layers of nodes in a directed graph, all of which are connected to each other. For data that cannot be separated in a linear fashion, it modifies the normal perceptron algorithm. It is possible to combine the compactness, moments, and Fourier descriptors for contours in training sets in neural network input values [19]. There are many advantages to using a multilayer perceptron instead of a single-layer perceptron when it comes to classification.

A simplified Bayesian classifier learning phase collects texture, spectral, and statistical information from each input mammography and builds models of real MCs for use as training samples. One of the most commonly used statistical methods for classifying data is the Bayesian classifier. In order to construct a binary image, a binary 0 or 1 is allocated to pixels categorized as class, 1 (or MCs), and a binary 1 is applied to pixels classified as class, 2 (or MCs), respectively (or healthy breast tissue).

## 3. Methods

Breast cancer is a deadly disease. This section contains a framework and related methods for the detection of breast cancer.  Figure 1 contains an image processing and machine learning enabled framework for breast cancer. In this framework, a set of mammogram images is used as input data set. Then, to improve the quality of these images, image processing is performed using the CLAHE algorithm. CLAHE (contrast limited adaptive histogram equalization) technique is an improvization of basic histogram equalization technique. This helps in removing noise from images, and it also results in improving image quality. Next step in the framework is image segmentation. In this step, pixels are labeled; it divides an image into different segments. This helps in locating objects and boundaries. These preprocessed images are classified using fuzzy SVM, Bayesian classifier, and random forest techniques.

The article "Effective Image Processing and Segmentation-Based Machine Learning Techniques for Diagnosis of Breast Cancer" was retracted in 2023. Reasons: signs of a paper mill; suspected computer-generated content; unreliable results or conclusions; concerns about the data.

For an image to be properly identified, the method used to extract the background must be able to adapt itself to match the unique features of a given image. In CLAHE, the histogram is only made for the pixel's surroundings. By setting a maximum, or “clip level,” to the height of the local histogram and thus the maximum contrast enhancement factor, CLAHE limits the maximum contrast adjustment that can be made. This reduces the amount of noise in the image at the end. CLAHE is better at making small parts of mammography look better [11]. When seen against a white background, the lesions are very clear. Even though this method makes it easier to see both signal and noise, there is still a lot of graininess in the photos.

The categorizing approach can be used in either a supervised or a specifically unsupervised manner. This is well established. Because of this, support vector networks are considered supervised machine learning standards. It is possible to define feature points or attribute states in terms of nonlinear hyperplanes and planar projections using an SVM [18]. The use of SVM is greatly influenced by factors such as the use of Gaussian kernels, the variance and standard deviation of the data, and the methods used to pick the kernels. Each training point in fuzzy SVM corresponds perfectly to a single class. The SVM was unable to classify any foci that are experiencing an eruption. In this way, FSVM is used to keep track of them. Data of a stochastic and probabilistic type necessitate prelearning data on the data sets themselves. Stochastic relationships can be identified in this section.

Factual and probabilistic data are used to create metadata in these types of classifiers. Bayes hypothesis (H) is employed with simple freedom guesses as one of the highlights in this example. It has been under constant scrutiny since the 1950s. It can be used for a variety of things, including medical diagnosis investigation, geographical imaging data, and content organization. In terms of changeable indicators, this classifier is quite versatile and requires a wide range of parameters. [20, 21]

Random forest may help with both classification and regression problems. The training step generates a huge number of decision trees, and each tree's outputs are predicted using regression algorithms. It has a low standard deviation, which makes it good for forecasting, and it connects different parts of the data rapidly. Random forest categorization was first met with skepticism by the general public since it is difficult to comprehend. However, in a prediction task, it has done better [21].

The article "Effective Image Processing and Segmentation-Based Machine Learning Techniques for Diagnosis of Breast Cancer" was retracted in 2023. Reasons: signs of a paper mill; suspected computer-generated content; unreliable results or conclusions; concerns about the data.

## 4. Results and Discussion

There are 322 images of the right and left breasts from mammograms in the MIAS database [22], which can be found here. There were 322 images in total, 51 of which were found to be malignant, 64 of which were found to be benign, and 207 of which were discovered to be normal. 250 images were used for the training of machine learning techniques, and remaining 72 images were used for the testing of classification techniques. First, images are preprocessed using the CLAHE algorithm, which is a variation of the CLAHE algorithm. Then, using the *K*-means algorithm, the images are segmented and analyzed. Preprocessing helps to remove noise from images, and segmentation aids in the detection of objects and boundaries in images. The images are then classified using techniques such as fuzzy SVM, Bayesian classifier, and random forest to determine their classification.

Five parameters, accuracy, sensitivity, specificity, precision, and recall, are used in experimental analysis.

(1) $$\begin{array}{c} \text{Accuracy}=\frac{\left(\text{TP}+\text{TN}\right)}{\text{TP}+\text{TN}+\text{FP}+\text{FN}}, \end{array}$$

(2) $$\begin{array}{c} \text{Sensitivity}=\frac{\text{TP}}{\text{TP}+\text{FN}}, \end{array}$$

(3) $$\begin{array}{c} \text{Specificity}=\frac{\text{TN}}{\text{TN}+\text{FP}}, \end{array}$$

(4) $$\begin{array}{c} \text{Precision}=\frac{\text{TP}}{\text{TP}+\text{FP}}, \end{array}$$

(5) $$\begin{array}{c} \text{Recall}=\frac{\text{TP}}{\text{TP}+\text{FN}}, \end{array}$$

where TP is true positive, TN is true negative, FP is false positive, and FN is false negative.

The confusion matrix is shown below in Table 1.

The accuracy, sensitivity, specificity, precision, and recall of different machine learning algorithms are shown below in Figure 2. The fuzzy SVM algorithm is performing better on all the comparison parameters.

## 5. Conclusion

People who have breast cancer are more likely to be women, but it can also happen to men, too. Only a few small differences separate the male and female breasts in structure. Anyone who wants to avoid breast cancer cannot do so with any method that is now available. Patients who are diagnosed and treated for breast cancer at an early stage have a better chance of having a successful treatment and recovery if they are taken care of quickly. It is widely agreed that digital mammography is a very good way to find breast cancer in its early stages. We may be able to use image processing techniques to detect breast cancer more quickly, which could help us both live and get better treatment. This article talks about a breast cancer image processing and machine learning system that was made. An example of input data for this framework is a set of mammography images. These images are used as input data. Images are then processed to make them look better by using the CLAHE method. This helps to remove noise from photos while also making the pictures better. There is still a lot of work to be done to the framework before it can start splitting images. Because the pixels are labeled at this point, an image is split into separate parts. This helps with the identification of objects and the drawing of boundaries. Techniques like fuzzy SVM, Bayesian classifier, and random forest are used to group these preprocessed images into groups. Five parameters, accuracy, sensitivity, specificity, precision, and recall, are used in experimental analysis. Fuzzy SVM is performing better than Bayesian classifier and random forest algorithm.

The article "Effective Image Processing and Segmentation-Based Machine Learning Techniques for Diagnosis of Breast Cancer" was retracted in 2023. Reasons: signs of a paper mill; suspected computer-generated content; unreliable results or conclusions; concerns about the data.

## Figures and Tables

**Figure 1:** Methodology for the classification and detection of breast cancer.

**Figure 2:** Accuracy, specificity, sensitivity, precision, and recall of classifiers for breast disease detection.

**Table 1:** Confusion matrix for breast cancer image classification.

Parameter	RF	KNN	LS-SVM-RBF
TP	161	174	197
TN	99	107	116
FP	32	23	4
FN	30	18	5

## Data Availability

The data shall be made available on request.
